# Towards malaria elimination in the MOSASWA (Mozambique, South Africa and Swaziland) region

**DOI:** 10.1186/s12936-016-1470-8

**Published:** 2016-08-18

**Authors:** Devanand Moonasar, Rajendra Maharaj, Simon Kunene, Baltazar Candrinho, Francisco Saute, Nyasatu Ntshalintshali, Natashia Morris

**Affiliations:** 1 Malaria Directorate, National Department of Health, Pretoria, South Africa; 2 Medical Research Council, Durban, South Africa; 3 National Malaria Programme, Ministry of Health, Manzini, Swaziland; 4 National Malaria Programme, Ministry of Health, Maputo, Mozambique; 5 Centro de Investigação em Saúde de Manhiça, Maputo, Mozambique; 6 Clinton Health Access Initiative, Manzini, Swaziland

**Keywords:** Malaria, Cross-border, Southern Africa, Elimination

## Abstract

The substantial impact of cross-border collaborative control efforts on the burden of malaria in southern Africa has previously been demonstrated through the successes of the Lubombo Spatial Development Initiative. Increases in malaria cases recorded in the three partner countries (Mozambique, South Africa, Swaziland) since termination of that programme in 2011 have provided impetus for the resuscitation of cooperation in the form of the MOSASWA malaria initiative. MOSASWA, launched in 2015, seeks to renew regional efforts to accelerate progress towards malaria elimination goals already established in the region. National malaria programmes, together with developmental partners, academic institutions and the private sector seek to harmonize policy, strengthen capacity, share expertise, expand access to elimination interventions particularly amongst migrant and border population groups, mobilize resources and advocate for long-term funding to ultimately achieve and sustain malaria elimination in the MOSASWA region.

## Background

Cross-border malaria control initiatives are important to supporting malaria elimination efforts, especially when low transmission countries share borders with higher transmission countries. The World Health Organization (WHO) Global Technical Strategy (GTS) 2016–2030 [1] and the Roll Back Malaria Action and Investment (AIM) Strategy 2016–2030 [2] advocate for cross-border collaboration to achieve successful malaria control and elimination. In southern Africa, Swaziland and South Africa, both low transmission countries, are pursuing the goal of malaria elimination by 2020 [3, 4]. South Africa and Swaziland share borders with Mozambique, a country that has a considerably higher burden of malaria [5]. The MOSASWA initiative aims to renew regional collaboration between Mozambique, South Africa and Swaziland.

The MOSASWA region consists broadly of eastern Swaziland, the southern Mozambican provinces of Maputo, Gaza and Inhambane, and the north-eastern districts of the South African provinces of KwaZulu-Natal, Mpumalanga and Limpopo (Fig. 1). The region constitutes approximately 14 % of the total land area of the three countries of 2,039,991 sq km. All 27.2 million of the inhabitants of Mozambique are at risk of malaria, compared with 28 % (356,077) in Swaziland and 10 % (5.4 million) in South Africa [5]. The parasite responsible for the majority of infection in the three countries is *Plasmodium falciparum*, with *Plasmodium malariae* and *Plasmodium ovale* also occurring in Mozambique. *Anopheles arabiensis* and *Anopheles funestus* represent the primary vectors in all three countries [6].

**Fig. 1:** The MOSASWA region consists of: Swaziland; the southern Maputo, Gaza and Inhambane provinces of Mozambique; and the malaria endemic districts of KwaZulu-Natal, Limpopo and Mpumalanga provinces of South Africa

Transmission in South Africa and Swaziland is seasonal, peaking between November and April, and is unstable and epidemic prone, but is stable and year-round in Mozambique.

Baseline incidence rates of 2.64 cases per 1000 population at risk in South Africa, 2.34 in Swaziland and 219 in Mozambique were recorded in 2014 at the commencement of the MOSASWA initiative [7]; however, incidence rates in Mozambique ranged between 0.01 and 500 at sub-district level, higher rates concentrated in the northern provinces and with substantially lower rates observed in the south [8]. Malaria is responsible for 29 % of all deaths and 42 % of deaths in children aged under 5 years in Mozambique, rendering it the most significant public health threat nationally [9]. Following the relative decline in national malaria incidence rates in Mozambique between 2007 and 2012, significant increases were recorded subsequently, rising from just over three million in 2013 to 5.5 million by 2014 (Fig. 2).

**Fig. 2:** Number of confirmed malaria cases reported in South Africa, Swaziland and Mozambique, 1982–2014

Mozambique has traditionally not implemented widespread indoor residual spraying (IRS) due to financial and logistical challenges, and has also prioritized its resources for the higher transmission and more populous north. Conversely, South Africa and Swaziland have invested heavily in the scale-up of IRS towards the goal of zero local transmission [10, 11]. However, the lack of coordinated regional efforts in this regard results in continued importation into the elimination areas. The MOSASWA initiative will jointly support the expanded coverage of a robust, efficiently executed IRS programme in Maputo Province, strengthen entomological surveillance and scale-up drug-based parasite clearance strategies towards transitioning the south to elimination.

The MOSASWA initiative is being built on the foundations of the Lubombo Spatial Development Initiative (LSDI), established in 1999 to address the issue of high malaria transmission in an area targeted for accelerated agricultural and economic development [6]. The primary emphasis of the LSDI malaria programme was to extend malaria control to southern Mozambique. There was increasing consensus that even if malaria control measures were optimal in South Africa and Swaziland (with effective treatment and insecticides in place), the disease burden could only be further reduced by a regional approach to control. The objectives of the LSDI were to: reduce malaria incidence in the border areas of South Africa and Swaziland from 250/1000 to fewer than 20/1000; reduce malaria infections from 625/1000 to fewer than 200/1000 within three years of commencement of IRS in Maputo Province; develop a regional malaria control programme to cover 200,000 sq km; develop a regional geographic information system (GIS)-based malaria information system (MIS) in the three countries; and, establish effective treatment and definitive diagnosis through the roll-out of rapid diagnostic tests (RDTs) and artemisinin-based combination therapy (ACT) at all public health facilities. The objectives of the LSDI malaria control initiative were realised within five years of initial implementation [12]. The initiative terminated in 2011 as the result of financing constraints. The substantial decline in the malaria burden realised during that period greatly improved the health quality of the targeted populations, and as a result, contributed to economic productivity in the region [13].

An increase in the burden of malaria in all three countries has been noted since the closure of the LSDI in 2011, despite sustained in-country implementation of malaria interventions in South Africa and Swaziland. Comparison of case counts recorded at baseline prior to the implementation of the LSDI (1999) with those observed at project termination in 2011 and again in 2014 just prior to the establishment of MOSASWA, reveals that gains achieved by the LSDI have been eroded subsequent to project termination in 2011 [5]. Consequently, resuscitation of cross-border collaboration is essential to return the malaria trend in the region to a downward trajectory.

Following the successes recorded by the LSDI, the impact of cross-border collaboration on regional malaria burden has been recorded through several other international initiatives, including the 13-country Asia-Pacific Malaria Elimination Network (APMEN) established in 2009 [14], the 11-country Amazon Malaria Initiative launched 2001 [15], and the Trans-Kunene Malaria Initiative between Namibia and Angola [16]. Capacity building, knowledge sharing, technical collaboration, sustainable financing, advocacy and political support have proven essential elements in the successful execution of all of these initiatives.

The MOSASWA malaria initiative has received political support from each of the participating countries through the signing of a declaration committing them to tackling malaria, particularly in the shared border areas of each country [17]. The goal of the initiative is to accelerate the transition from pre-elimination to elimination of malaria in Swaziland and South Africa, and from control to pre-elimination in southern Mozambique, so as to achieve zero local transmission in Swaziland, South Africa and Maputo Province (Mozambique) by 2020 and achieve pre-elimination status in Gaza and Inhambane provinces (Mozambique) by 2025 [18]. Key objectives are to: (1) harmonize policies, strengthen sub-national capacities and share expertise; (2) expand access to malaria elimination interventions with particular focus on mobile and migrant populations, malaria risk localities and residents to reduce and interrupt malaria transmission; (3) strengthen capacity for surveillance, operational research and monitoring and evaluation; and, (4) mobilize resources and advocate for increased long-term financing to achieve and sustain malaria elimination across the MOSAWA region.

Some 18 key strategies are identified under the four objectives outlined in the MOSASWA Strategic Plan 2016–2020 [7]. Broadly these are to: engage with state leadership to champion the regional elimination agenda; strengthen regional leadership towards a coordinated cross-border elimination approach; strengthen and harmonize vector control, entomology, information sharing, surveillance, guidelines and policies; understand and map regional transmission pathways and foci; strengthen health service delivery in border areas; implement operational research to create the necessary knowledge to inform regional strategy; mobilize resources and advocate for increased and sustainable financing to achieve malaria elimination; explore innovative financing mechanisms; promote private sector engagement in the initiative; and, seek government advocacy to increase domestic malaria funding allocation.

The MOSASWA initiative is built on the solid foundation of the LSDI, from which capacity still exists in all three affected countries for implementation of strategies and management of the initiative. Although malaria cases in the MOSASWA region increased in the 2012–2015 period, numbers remain relatively low. Every effort needs to be made to reverse the recent trend, to bring these areas back onto the elimination trajectory.

Financing required for the MOSASWA initiative to implement its 2016–2020 strategic plan is in the region of 39 million US$. Funding for this initiative, albeit challenging, will need to be sourced via domestic financing mechanisms to ensure sustainability.

MOSASWA forms part of the broader Elimination Eight (E8) malaria initiative consisting of collaboration amongst eight southern African countries. The goal of the E8 initiative is to enable and accelerate toward zero local transmission in the four front-line countries (Botswana, Namibia, South Africa, Swaziland) by 2020 and achieve the same in the second-line countries (Angola, Mozambique, Zambia, Zimbabwe) by 2030 [19]. Regional coordination and management, securing and sustaining political support, enabling cross-border programming and resource mobilization are the five key objectives of the E8 initiative. The MOSASWA initiative is directly aligned to the goals and strategies of the E8. Moreover, mobilization of funds may be leveraged using the E8 as a parent initiative.

Each of the three partner countries is pursuing aggressive malaria control and elimination interventions with the common eventual goal of eliminating malaria. Specific challenges exist within each country’s individual borders, varying with the respective epidemiology, intrinsic receptivity, and funding landscape of each, and successful elimination will require efforts across all programme areas. Many of these challenges will need to be met by the individual countries. However, malaria transmission dynamics amongst these countries are highly connected and interdependent, being linked through population movement and malaria ecologies. Hence, it is in the collective best interest to operationalize cross-border collaboration to reduce the impact and burden of malaria locally and trans-nationally. The MOSASWA initiative will require that best practices and lessons learnt from the LSDI be effectively applied in order to assure a sustained long-term effort wholly owned by the MOSASWA countries.

The MOSASWA initiative comes at an important stage in the malaria elimination efforts of Swaziland and South Africa. For these two countries to have a realistic chance at elimination, neighbouring Mozambique’s collaboration will be pivotal. Further, escalation of control efforts in Maputo Province will ensure its own accelerated transition towards elimination.

Over the past decade, all three participant countries have achieved substantial reductions in their malaria burden. In South Africa and Swaziland, malaria is now limited to border districts and malaria cases among migrant populations represent a high proportion of the total number of recorded cases. Mobile populations pose the greatest challenge to achieving malaria elimination. As has been observed post-termination of the LSDI, movement of people from high-transmission areas to areas with very low transmission results in an increase in the number of malaria cases in the host country or region. Progress towards malaria elimination in these countries will require improved access to health services for these groups. As the southern African region moves towards malaria elimination, ministries of health need to ensure that migrants, refugees and mobile populations have adequate access to prevention interventions as well as prompt diagnostics and effective treatment. This ideal is enshrined within the MOSASWA strategic plan.

## Conclusion

The MOSASWA initiative is an adjunct to country pre-elimination and elimination efforts. Swaziland and South Africa’s reduced malaria case numbers places these countries firmly in the elimination and pre-elimination phases, respectively, however it is imperative that malaria interventions are optimized across their borders with Mozambique to give these countries a real chance at elimination of the disease. Whilst migration and cross-border movement of persons is a direct focus area of MOSASWA, in-country activity will not diminish. Surveillance, screening and treatment, together with effective vector control, will be the key drivers to removing malaria reservoirs in eliminating countries. The most serious threat to malaria elimination is not resurgence due to insecticide or drug resistance, but non-implementation of effective interventions due to non-sustainable funding. Sustained, adequate funding is necessary to maintain the gains made in the control phase and access to increased funding is necessary as countries progress towards elimination. As evidenced post termination of the LSDI, gains achieved over decades can be eroded in a matter of months when preventative and curative processes deteriorate. The MOSASWA initiative, through sound political commitment, is pursuing funding for the start-up phase of the first 3 years. Thereafter, it is up to domestic funding together with private–public partnerships to warrant that the initiative is well funded and that the gains made in the fight against malaria are maintained through to elimination [9]. The MOSASWA initiative must maintain the gains made through the initial international investment by mobilizing and maintaining adequate levels of funding, political commitment and strong operational capacity in all countries to continue using effective tools as part of a co-ordinated regional effort [20]. Notwithstanding this, human resource capacity needs to be built and maintained to ensure that control and elimination efforts of the MOSASWA initiative remain on track.

## Abbreviations

WHO: World Health Organization
GTS: Global Technical Strategy
AIM: Roll Back Malaria Action and Investment Strategy
IRS: indoor residual spraying
LSDI: Lubombo Spatial Development Initiative
GIS: geographic information system
MIS: malaria information system
ACT: artemisinin-based combination therapy
RDT: rapid diagnostic test
APMEN: Asia–Pacific Malaria Elimination Network
E8: Elimination Eight Malaria Initiative
